The article "Genome-wide analysis of bZIP, BBR, and BZR transcription factors in Triticum aestivum" was retracted in 2022. Reasons: compromised peer review; a conflict of interest; concerns about the authorship.

# Genome-wide analysis of bZIP, BBR, and BZR transcription factors in *Triticum aestivum*

**DOI:** 10.1371/journal.pone.0259404

**Published:** 2021-11-30

**Authors:** Arzoo Ahad, Roohi Aslam, Alvina Gul, Rabia Amir, Faiza Munir, Tuba Sharf Batool, Mahnoor Ilyas, Muhammad Sarwar, Muhammad Azhar Nadeem, Faheem Shehzad Baloch, Sajid Fiaz, Muhammad Abu Bakar Zia

**Affiliations:** 1 Department of Plant Biotechnology, Atta-ur-Rahman School of Applied Biosciences, National University of Sciences and Technology, Islamabad, Pakistan; 2 NUTECH School of Applied Sciences and Humanities, National University of Technology, Islamabad, Pakistan; 3 National Institute for Biotechnology and Genetic Engineering (NIBGE), Faisalabad, Pakistan; 4 Faculty of Agricultural Sciences and Technologies, Sivas University of Science and Technology, Sivas, Turkey; 5 Department of Plant Breeding and Genetics, The University of Haripur, Hyber Pakhtunkhwa, Pakistan; 6 College of Agriculture, Bahauddin Zakariya University, Bahadur sub–Campus Layyah, Punjab, Pakistan; Anhui Agricultural University, CHINA

## Abstract

Transcription factors are regulatory proteins known to modulate gene expression. These are the critical component of signaling pathways and help in mitigating various developmental and stress responses. Among them, bZIP, BBR, and BZR transcription factor families are well known to play a crucial role in regulating growth, development, and defense responses. However, limited data is available on these transcription factors in *Triticum aestivum*. In this study, bZIP, BBR, and BZR sequences from *Brachypodium distachyon*, *Oryza sativa*, *Oryza barthii*, *Oryza brachyantha*, *T*. *aestivum*, *Triticum urartu*, *Sorghum bicolor*, *Zea mays* were retrieved, and dendrograms were constructed to analyze the evolutionary relatedness among them. The sequences clustered into one group indicated a degree of evolutionary correlation highlighting the common lineage of cereal grains. This analysis also exhibited that these genes were highly conserved among studied monocots emphasizing their common ancestry. Furthermore, these transcription factor genes were evaluated for envisaging conserved motifs, gene structure, and subcellular localization in *T*. *aestivum*. This comprehensive computational analysis has provided an insight into transcription factor evolution that can also be useful in developing approaches for future functional characterization of these genes in *T*. *aestivum*. Furthermore, the data generated can be beneficial in future for genetic manipulation of economically important plants.

## Introduction

Plants, being sessile organisms, have established multiform signalling pathways for protection against several biotic factors such as microbes, insects, weeds, and abiotic factors such as drought, salinity, and extreme temperature [1]. Transcription factors (TFs), being an important regulator, help to modulate gene transcription in response to environmental cues in the form of pattern triggered immunity (PTI) and effector-triggered immunity (ETI). Pathogenic Microbe-Associated Molecular Patterns induce PTI (MAMPS) recognized by plant cell surface receptors conferring transient response [2]. ETI is associated with the release of effectors molecules of microbes identified by the R-proteins [3]. These induce a prolonged immune response by activating reactive oxygen species (ROS) and TFs [4]. They help trigger the gene expression and level of transcription by binding to the regulatory DNA within the targeted gene [5]. There are 58 TFs present in plants to activate and repress a particular gene’s expression pattern [6]. Six of them significantly contribute to gene regulation viz., bZIP, WRKY, BHLH, AP2/ERF, MYB, and NAC transcription factors [7].

The article "Genome-wide analysis of bZIP, BBR, and BZR transcription factors in Triticum aestivum" was retracted in 2022. Reasons: compromised peer review; a conflict of interest; concerns about the authorship.

Among these plant TFs, one of the significant and dissimilar transcription factor families in developed plants is the basic leucine zipper (bZIP) [8]. The various numbers of bZIP genes were identified in plants ranging from 89 in *Oryza sativa* [9], 92 in *Sorghum bicolor* [10], 187 in *Triticum aestivum* [11], 125 in *Zea mays* [12], 69 in *Solanum lycopersicum* [13], 75 in the case of *Arabidopsis thaliana*, and 49 in *Ricinus communis* [14]. They possess a bZIP domain (40–80 amino acids in length) comprising of basic and leucine zipper region [15]. In plants, bZIP TFs are documented to have a significant role in regulating growth, sexual development, sugar, and hormonal signaling, microbial pathogen defense, cell elongation, and metabolism regulation. A considerable number of bZIP TFs are characterized in Arabidopsis; for example, *At*bZIP*17* and *At*bZIP*24*. In *O*. *sativa* role of some of the bZIP genes have also been studied in detail. For instance, OsbZIP16, OsbZIP23, and OsbZIP72 are reported as constructive regulators for drought stress. Another *Os*bZIP*60* is registered to be regulated by drought as well as heat [11]. Another transcription factor family is Barley B recombinant (BBR), which is still poorly characterized. They derive their name from a highly conserved BPC domain located at C-terminal [16]. This domain has a greater degree of sequence analogy and is evolutionarily conserved. In plants, members of BBR have been reported as developmental regulators. They also have a distinctive role in auxin, cytokinin, and ethylene signalling [17]. There are three classes of BBR/BPC genes; class I (BPC1- BPC3), class II (BPC4- BPC6, class III (BPC7) [18] based on the diversity of N- terminus [19]. BRASSINAZOLE-RESISTANT (BZR) is a plant-specific transcription factor that regulates Brassinosteroids (BR) signalling. Brassinosteroids targets BZR by binding to a membrane-localized receptor, BRASSINOSTEROID-INSENSITIVE 1 and control genes of BR signalling. BRs are involved in cell elongation, vascular differentiation, senescence, and photomorphogenesis, protecting plants from various environmental cues. In *Arabidopsis thaliana*, AtBZR1 regulates freezing tolerance through dehydration-responsive element-binding protein (DREB) dependent independent pathways [20]. In rice, *OsBZR* family has a conserved role similar to that of *Arabidopsis*. In *T*. *aestivum*, *TaBZR2* serves as a positive regulator of drought tolerance [21].

The article "Genome-wide analysis of bZIP, BBR, and BZR transcription factors in Triticum aestivum" was retracted in 2022. Reasons: compromised peer review; a conflict of interest; concerns about the authorship.

Although transcription factors such as bZIP, BBR, and BZR play a significant role in plant development. However, to date, no significant information is available in *T*. *aestivum*. It is crucial to understand the exact evolutionary origins of TabZIPs, TaBBRs, and TaBZRs and their roles in stress biology. Based on this, the current project aims to provide a detailed computational analysis of bZIP, BBR, and BZR transcription factors in *T*. *aestivum* to provide insight for future strategies for functional analysis such as seed germination, growth of seedlings, high temperature and cold tolerance, to name a few. To conduct this research work, *B*. *distachyon* was used a model plant. In the post genomics era, the *B*. *distachyon* is a model system that enhances our understanding of the biology of grasses, especially tiny grains. It is the developing model plant of the Poaceae family. It has become more significant in applied functional genomics because of its great competence for genetic manipulation and compact genome. Its research is progressing quickly, with topics such as grain growth, starch accumulation, biofuel production, biotic and abiotic stress responses [22]. Comparison of the genomes of genus *Brachypodium*, *Oryza*, and *Sorghum* uncovers a detailed history of genomic evolution across a wide range of grasses and offers a framework for studying the massive genomes of commercially significance grasses like *T*. *aestivum* [23]. Furthermore, phylogenetic, and conserved motif analyses were accomplished to discover the evolutionary relationship among different Poaceae species. Gene structure was predicted to obtain a clear depiction of the number and position of the exon/intron. Subcellular localization of TabZIP, TaBBR, and TaBZR proteins were confirmed. The information can be beneficial in future for further wet-lab experiments for genetic manipulation of economically important plants.

The article "Genome-wide analysis of bZIP, BBR, and BZR transcription factors in Triticum aestivum" was retracted in 2022. Reasons: compromised peer review; a conflict of interest; concerns about the authorship.

## Material and methods

### Sequence retrieval and identification of bZIP, BBR, and BZR proteins

Sequences of bZIP, BBR, and BZR transcription factors families from 8 species (*B*. *distachyon*, *O*. *sativa subsp*. *japonica*, *O*. *brachyantha*, *O*. *barthii*, *T*. *aestivum*. *T*. *urartu*. *Z*. *mays*, and *S*. *bicolor*) were selected for this research. *B*. *distachyon* was used as a model, and its annotated bZIP, BBR, and BZR protein sequences were identified and retrieved from *B*. *distachyon*. Genome Database (BdGDB) [24] with designated name. These sequences were also verified through locus ID’s present on Grassius [25]. *B*. *distachyon* bZIP, BBR, and BZR sequences served as a query to search for *O*. *sativa subsp*. *japonica*, *O*. *brachyantha*, *O*. *barthii*, *T*. *aestivum*. *T*. *urartu*. *Z*. *mays*, and *S*. *bicolor* by Blastp analysis in UniprotKB [26], NCBI [27] and Ensemble plants [28].

### Phylogenetic analysis and multiple sequence alignment

ClustalW was used to perform Protein sequence alignment [29] and MEGA X was used for phylogenetic analysis (Version 10.2.2) [30] using Maximum likelihood method founded on JTT matrix-based model [31] using default parameters.

### Motif analysis of TabZIP, TaBBR, and TaBZR proteins

Identification of conserved domain was performed by Clustal Omega [32] and alignment file was presented in Genedoc [33]. Additional conserved protein motifs outside bZIP, BBR and BZR domain was also screened using MEME tool [34]. The descriptors limit used for carrying out motif analysis was specified as follows: Number of motifs: 15 (bZIP), 8 (BBR), and 5 (BZR), Least motif width: 6, Extreme motif width: 50, Distribution of motif sites: 0 or 1/ sequence.

### Identification of subcellular localization and gene structure of TabZIP, TaBBR, and TaBZR protein

The bZIP, BBR, and BZR subcellular localization for *T*. *aestivum* were predicted by freely accessible tool Plant-mPLoc [35]. Besides plant-mPLoc, ‘LOCALIZER’ [36] was also used to predict the localization of plant proteins in different cell compartments. The gene structure of bZIP, BBR, and BZR for *T*. *aestivum* were mapped using the CDS and genomic sequences. The exon/intron organization was determined and demonstrated employing the Gene Structure Display Server (GSDS2.0 platform) [37].

## Results

### Sequence retrieval and phylogenetic analysis

Full-length sequences for three transcription factors families from eight monocotyledonous plants were retrieved from different databases. The detail of proteins including, accession number, amino acid sequence length, and databases are given in S1–S3 Tables.

The article "Genome-wide analysis of bZIP, BBR, and BZR transcription factors in Triticum aestivum" was retracted in 2022. Reasons: compromised peer review; a conflict of interest; concerns about the authorship.

### bZIP Phylogenetic tree

The phylogenetic tree (Fig 1**)** composed of 662 amino acid sequences (S1 Table) was clustered in two major branches. The two major branches were further divided into clades and subclades. Each clade was formed of one gene sequence from various species. The clade names were given based on the *B*. *distachyon* bZIP gene number (bZIP1 to bZIP85). It was speculated that the bZIP clustered into one group, might show a greater degree of relatedness highlighting the common ancestry of Poaceae. Phylogenetic analysis showed that the clade size of each bZIP gene is not the same indicating that number of bZIP genes in each plant varied.

**Fig 1:** Phylogenetic analysis using Maximum Likelihood method. The tree with the superior log likelihood (-173413.62) is shown in the figure. The analysis of bZIP involved 662 amino acid sequences. There were a total of 1890 positions in the final dataset.

For bZIP26 and bZIP84 genes, one homeolog for *T*. *aestivum* i.e.,5A and 2A were reported respectively in the searched databases. The other two homeologs B and D for both bZIP genes were not found. The bZIP27, bZIP62, and bZIP72 clades did not contain the B genome of *T*. *aestivum* whereas two homeologs A and D were found. Two homeologs 1A and 1B were found for bZIP35 but the third D homeolog was missing. Phylogram indicates that the bZIP42 clade consist of D genome of *T*. *aestivum*. Homeologs A and B were missing in this clade.

#### BBR phylogenetic tree

The BBR tree was shaped using amino acid sequences of full-length from all eight plants. The final tree involved 17 amino acid sequences (S2 Table). The tree was diverged into two clades BBR1 and BBR2 shaded in green and red color, respectively (Fig 2**)**. The monocotyledonous plants that fall in the same clade represented the same ancestry of BBR transcription factor. In the case of the Poaceae family, BBR genes are not well studied. The BBR1 clade has all the eight species except the B and D homologue of *T*. *aestivum*. BBR2 clade is also composed of all species except *T*. *urartu* however A homeolog of *T*. *aestivum* is present in this clade.

**Fig 2:** Phylogenetic analysis using the Maximum Likelihood method. The tree with the superior log likelihood (-4765.88) is shown. The analysis of BBR involved 17 amino acid sequences. There was a total of 479 positions in the final dataset.

#### BZR phylogenetic tree

There were seven clades in the final phylogenetic tree from BZR1 to BZR7 (Fig 3) ranging from 67–715 amino acid length. The final tree involved 56 amino acid sequences (S3 Table). BZR1 clade was short of only *T*. *urartu* sequence but the A genome of *T*. *aestivum* is present in this clade. *Z*. *mays* and *S*. *bicolor* lie near each other in the tree and these were not present in the clade of BZR2. BZR6 clade was composed of three monocotyledonous while *O*. *sativa*, *O*. *brachyantha*, *O*. *barthii*, *T*. *aestivum*, *T*. *urartu* were missing. All the clades were found of three homeolog of each *T*. *aestivum* gene except BZR6 and BZR5. Interestingly, the *T*. *urartu* sequence was also absent in BZR6 clade which is a close relative of *T*. *aestivum* and adds A genome to it providing an evolutionary history of *T*. *aestivum*.

The article "Genome-wide analysis of bZIP, BBR, and BZR transcription factors in Triticum aestivum" was retracted in 2022. Reasons: compromised peer review; a conflict of interest; concerns about the authorship.

**Fig 3:** Phylogenetic analysis using the Maximum Likelihood method. The tree with the superior log likelihood (-17893.92) is shown. The analysis of BZR involved 56 amino acid sequences. There was a total of 920 positions in the final dataset.

### Conserved motif analysis of *T*. *aestivum*

#### Motif analysis of bZIP for *T*. *aestivum*

To confirm the presence of basic (N-X7-R/K) and leucine zipper domain (L-X6-L-X6-L) alignment of bZIP proteins were performed by Clustal Omega and the results were visualized in Genedoc. The results confirmed the presence of conserved bZIP domain (S1A–S1D Fig) The occurrence of surplus preserved motifs outside the domain of bZIP was also confirmed from a set of 196 *T*. *aestivum* protein sequences between 149 and 652 in length using MEME software (S2 and S3A–S3E Figs).

#### Motif analysis of BBR/BPC for *T*. *aestivum*

For the identification of conserved BBR/BPC domain sequence alignment was done. It was noticed that there were three highly conserved regions (Fig 4). First, five conserved cysteine residues. Second, RxxGRKMS motif. Third, the WAKHGTN region. A highly conserved TIR motif was also observed parallel to WAKHGTN. The presence of additional conserved motif other than the BBR/BPC domain was confirmed from a set of four protein sequences between 331 and 349 in length (average length 343.5) using MEME software. The logo (S4A Fig) and the location (S4B Fig) of the conserved motif were predicted. It was noted that motifs 1 and 2 were conserved in all the 4 *T*. *aestivum* protein sequences.

**Fig 4:** Conserved domain analysis of BBR/BPC.

#### Motif analysis of BZR for *T*. *aestivum*

Conserved motifs from 15 protein sequences between 178 and 686 in length (average length 366.7) were identified by MEME software and motif logos (S5A Fig) and locations (S5B Fig) were predicted. The results showed that motif 3 was found conserved in all 15 sequences.

### Identification of subcellular localization of T. aestivum bZIP, BBR, and BZR transcription factors

#### Subcellular localization of *T*. *aestivum* bZIP

According to localizer prediction (S6A, S6B and S6C Fig) most of the *T*. *aestivum* bZIP were nuclear-localized except three (TraesCS3B02G167500.1, TraesCS1B02G282800.1, and TraesCS1A02G273000.1) and according to Plant mPLoc prediction (S4 Table)., all the *T*. *aestivum* bZIP were localized in the nucleus except TraesCS7A02G511600.1 and TraesCS7D02G501500.1. The former was localized in the cell membrane and chloroplast while the later was chloroplast, cell membrane, and nuclear-localized.

The article "Genome-wide analysis of bZIP, BBR, and BZR transcription factors in Triticum aestivum" was retracted in 2022. Reasons: compromised peer review; a conflict of interest; concerns about the authorship.

### Subcellular localization of *T*. *aestivum* BBR

According to localizer (S7A Fig) and Plant mPLoc prediction all the BZR proteins possesses NLS and were localized in the nucleus.

#### Subcellular localization of *T*. *aestivum* BZR

According to localizer (S8 Fig) all the BZR proteins were localized in the nucleus except the A genome (TraesCS4A02G307900.1) of TaBZR7. mPLoc evaluation predicted that all BZR proteins were present in the nucleus (S6 Table).

### Gene model prediction of *T*. *aestivum* bZIP, BBR, and BZR

#### Gene model prediction of bZIP

To further understand the relationship of bZIP proteins, gene models were predicted using GSDS (S9A, S9B, S9C and S9D Fig). It was noted that in each bZIP gene the exons and introns vary. The maximum number of exons were 12 and the minimum number of exons was 1 (S4 Table). Moreover, intron-less *Ta*bZIP*s* were also present.

#### Gene model prediction of BBR

It was examined that there were three intron-less transcripts, and one transcript with only one intron. Exons number also varies with a least of one and a maximum of two in number (S7B Fig, S5 Table).

#### Gene model prediction of BZR

In *TaBZR*, there were twelve transcripts with one intron, two transcripts with seven introns, and only one transcript with eight introns (Fig 5). Overall, no transcript was intron-less. The number of introns ranged from two-eight. The number of exons varies from two to eight (S6 Table).

**Fig 5:** Gene model prediction of TaBZR.

## Discussion

Comparative genomics is playing a prominent role in obtaining effective data from biological sequences. Comparison of protein, gene order, and location from more than one organism is an important facet of comparative genomics. Such type of analysis helps in studying similarities, differences, and evolutionary biology. The availability of plant whole genome sequencing through NGS provides convenience in developing markers in addition to the identification of agronomically significant traits [38]. The availability of the sequenced genome of *A*. *lyrate*, *B*. *distachyon* [39], *A*. *thaliana* [40], *O*. *sativa* [41] provides opportunity for the explanation of other genomes of grasses. For many decades *A*. *thaliana* has been adopted as a model plant due to its short and rapid life cycle, small size, self-pollinating ability, and easily manipulatable genome [42]. *O*. *sativa* also serves as a model for cereal crops. Its genome is 400 Mb which is the smallest among cereals but 4 times larger than *A*. *thaliana*. Comparative genomics has remodeled the thinking that the genome of *O*. *sativa* can be used for the identification of other cereal genomes including *T*. *aestivum*, *Z*. *mays*, *S*. *bicolor* because of conserved synteny across their genomes [43]. Recently, it was reported that *B*. *distachyon* genome is more closely related to *T*. *aestivum* as compared to *O*. *sativa* [44]. It has all the attributes of a model plant such as small genome size (~355MBp), self-fertility, short life cycle (8–11 weeks), simple growth conditions, and easily manipulatable genome. Based on this, a similar pathway was utilized for the retrieval of the bZIP, BBR, and BZR sequences from different plants of the Poaceae family.

The article "Genome-wide analysis of bZIP, BBR, and BZR transcription factors in Triticum aestivum" was retracted in 2022. Reasons: compromised peer review; a conflict of interest; concerns about the authorship.

A phylogenetic tree with 662 members of bZIP family was constructed using the Maximum likelihood method. For bZIP26 and bZIP84 genes, B and D homeologs were not found in the databases. According to the established evidence, the contributor of the D-genome of *T*. *aestivum* is *A*. *taushii* [45] and the presenter of the B-genome is still under debate, but it is expected to be *A*. *speltoides*. A gene loss event might be happened resulting in the loss of these homeologs in *T*. *aestivum*. The clade for bZIP42 consists of the D genome of *T*. *aestivum* while the A as well as B homeologs were missing. *T*. *urartu* that is responsible for adding A genome to *T*. *aestivum* [46] is present in this clade. The reason for the missing of two homeologs in *T*. *aestivum* might be the uncharacterized protein sequences for *T*. *urartu* and *A*. *speltoides*. Only 48 clades have sequences for *T*. *urartu*, which is the diploid progenitor of the A genome in *T*. *aestivum*. The clade of bZIP1, bZIP6, bZIP13, bZIP39, bZIP56, bZIP57, bZIP59, and bZIP72 does not contain *T*. *urartu* as well as A homeolog of *T*. *aestivum* suggesting the possibilities that these genes may be under selection pressure and results in heightening the rate of protein evolution. The result of this analysis also indicates a close relation between *Z*. *mays* and *S*. *bicolor* because they lie close to each other in the phylogenetic tree. An earlier report also supports the presence of conserved syntenic regions between *Z*. *mays* and *S*. *bicolor* [43]. *Z*. *mays* and *S*. *bicolor* sequences appeared closely related to model plant rice as compared to *B*. *distachyon*. So, *O*. *sativa* sequences can help to annotate other sequences of *Z*. *mays* and *S*. *bicolor*.

The article "Genome-wide analysis of bZIP, BBR, and BZR transcription factors in Triticum aestivum" was retracted in 2022. Reasons: compromised peer review; a conflict of interest; concerns about the authorship.

The BBR phylogenetic tree was divided into two main sub clades. The BBR1 clade showed the absence of B and D homologue of *T*. *aestivum* that might be because of evolutionary events. *T*. *urartu* being the wild progenitor of A genome of *T*. *aestivum* is present in this clade along with A genome of *T*. *aestivum* supporting the fact that *T*. *Urartu* contributes A genome to *T*. *aestivum*. The monocotyledonous falling in the same clade represents the monophyletic relation of all monocots. BBR2 clade contains all the selected species except *T*. *urartu* however A homeolog of *T*. *aestivum* is present in this clade. The absence of *T*. *urartu* protein sequence indicated that the gene product might not be translated into protein transcript. *O*. *sativa* and *B*. *distachyon found* closely lying in both clades which showed syntey among grass species despite of fluctuations and evolutionary divergence in the genome size. The BZR phylogenetic tree was composed of seven clades. BZR1 clade showed the absence of only *T*. *urartu* sequence. *Z*. *mays* and *S*. *bicolor* lie in close proximity to each other in the tree and their absence in the BZR2 clade supports that they have close synteny that can be examined over comparative genomics [47]. There must be close functional and evolutionary acquaintance between *Z*. *mays* and *S*. *bicolor*. BZR6 and BZR5 clade showed irregularities. They do not have three genomes of *T*. *aestivum*. Interestingly, *T*. *urartu* sequence was also absent in the BZR6 clade which is a close relative of *T*. *aestivum*. The absence of *T*. *urartu* indicates the loss of genes during the process of recombination [48].

Alignment of bZIP proteins by Clustal Omega confirmed the occurrence of conserved bZIP domain in all the proteins. In addition to bZIP, a total of 14 motifs outside the bZIP domain were discovered by MEME tool. Additional motifs might be engaged in the proper functioning of bZIP proteins [1]. BBR/BPC conserved domain analysis results in the identification of five cysteine residues, RxxGRKMS motif, and WAKHGTN region. A highly conserved TIR motif parallel to WAKHGTN has also been noticed. The conserved WAR/KHGTN motif helps the BBR/BPC protein in binding to the DNA and DNA bending. This motif is comparable in amino acid length and composition of conserved WRKYGQK in WRKY proteins. A similar bending pattern for WAR/KHGTN in BBR/BPC was proposed as observed for WRKY [19]. Outside BBR domain additional motifs were also present. Conserved motifs from BZR protein sequences between 178 and 686 in length were identified by MEME software. The results showed that motif 3 was highly conserved in all 15 sequences. The conserved BZR region helps in DNA-binding because of the atypical bHLH DNA-binding motif [49]. Sub-cellular localization is important for the proper functioning of protein and achieving functional diversity [50]. Plant proteins translocating from cytosol to chloroplast and mitochondria require N-terminal transit peptides and nuclear localization signals (NLS) for nuclei [36]. Subcellular localization of *T*. *aestivum* bZIP, BBR, and BZR proteins predicted by LOCALIZER showed that out of 196 *T*. *aestivum* bZIP proteins, 3 proteins (1.5%) were with chloroplast localization and NLS and 192 (98.0%) with NLS and no transit peptides. The B genome of *T*. *aestivum* bZIP28 (TraesCS3B02G167500.1) has a probability of 0.752 for containing chloroplast transit peptide at position 1–72 with no localization signal for mitochondria but NLS (KRIIANRQSAQRSRVRKL, KRVKRIIANRQSAQRSRVR) is present. The B (TraesCS1B02G282800.1) and A (TraesCS1A02G273000.1) genome of *T*. *aestivum* bZIP35 have a probability of 0.961 for chloroplast transit peptide at 1–26 position with no mitochondrial localization. Most of the bZIP proteins showed NLS and were nuclear-localized. Earlier publications reported the presence of the N-x7-R/K-x9 motif for DNA-binding and nuclear localization [14, 51]. Reports on *A*. *thaliana* confirm the presence of bZIP on multiple locations i.e., ER and nucleus [52]. The in silico subcellular localization of all BBR proteins displayed 100% NLS and no transit peptides were present. They were localized in the nucleus. The transportation of TF in the nucleus is an active process. TF functions work efficiently in the nucleus. NLS is a short peptide sequence rich in Arginine and Lysine residues controlling the ingression of TF into the nucleus efficiently. Subcellular localization of TaBZR proteins indicated that 14 (93.3%) proteins were with NLS and no transit peptides. A genome of TaBZR7 (TraesCS4A02G307900.1) have no NLS. Earlier in silico subcellular localization prediction of *ZmBZR* reported that most of them were nuclear-localized [53]. Plant mPLoc predicts the location of proteins at the following sites: Cell wall, nucleus, vacuole, chloroplast, extracellular, cytoplasm, plasma membrane, endoplasmic reticulum, plastids, mitochondria, peroxisome [35]. According to Plant mPLoc prediction, all the TabZIPs were localized in the nucleus except A and D homeolog of TabZIP11. The A homeolog (TraesCS7A02G511600.1) exist in in the cell membrane and chloroplast. The D homeolog (TraesCS7D02G501500.1) exist in in the cell membrane, chloroplast along with the nucleus. According to plant mPLoc, all TaBBR and TaBZR were predicted to localize in the nucleus.

The article "Genome-wide analysis of bZIP, BBR, and BZR transcription factors in Triticum aestivum" was retracted in 2022. Reasons: compromised peer review; a conflict of interest; concerns about the authorship.

GSDS version 2.0 was used to predict exon/intron pattern of *Ta*bZIP, *TaBBR*, and *TaBZR*. The exon/intron pattern of each gene gives idea about its evolutionary relationship. It was noted that number of exons and introns vary in each. *Ta*bZIP*34*, *Ta*bZIP*45*, *Ta*bZIP*71*, and *Ta*bZIP*80* possess 12 exons that were highest among all the studied bZIP. The minimum number of exons was 1 noted from *Ta*bZIP*3*, *Ta*bZIP*4*, *Ta*bZIP*24*, *Ta*bZIP*31*, *Ta*bZIP*37*, *Ta*bZIP*38*, *Ta*bZIP*41*, *Ta*bZIP*49*, *Ta*bZIP*52*, *Ta*bZIP*60*, *Ta*bZIP*63*, *Ta*bZIP*66*, *Ta*bZIP*68*, and *Ta*bZIP*75*. Difference in intron number and position were also observed. *Ta*bZIP*4*, *Ta*bZIP*3*, *Ta*bZIP*10*, *Ta*bZIP*31*, *Ta*bZIP*37*, *Ta*bZIP*38*, *Ta*bZIP*24*, *Ta*bZIP*41*, *Ta*bZIP*49*, *Ta*bZIP*52*, *Ta*bZIP*60*, *Ta*bZIP*66*, *Ta*bZIP*68*, *Ta*bZIP*75*, and *Ta*bZIP*63* lack intron. The lack of intron might minimize the posttranscriptional mechanism for direct response to abiotic stress. In *TaBZR*, no intron-less transcript was observed. The number of exons varies from two to eight. It was noted that *TaBBR* were mostly intron-less except A genome of *TaBBR1* having one intron. The gain or loss of intron in genes may arise during the evolution of *TaBBR* genes [1].

## Conclusion

This is the first study that provides genome-wide, in-depth analysis of bZIP, BBR, and BZR transcription factors from eight plant species of the Poaceae family with notable consideration to *T*. *aestivum*. In this analysis, bZIP, BBR, and BZR gene families were subjected to phylogenetic analysis. Moreover, *T*. *aestivum* bZIP, BBR, and BZR genes were further explored for motif identification, gene structure and localization prediction. This comprehensive analysis demonstrated that these genes were highly conserved among different monocots highlighting their common ancestry. The study also showed that *B*. *distachyon* is phylogenetically closer to *T*. *aestivum*. Hence, *B*. *distachyon* can help to provide functional along with evolutionary knowledge to annotate genes in *T*. *aestivum*. Similarly, it was revealed that *Z*. *mays* and *S*. *bicolor* were closely related to *O*. *sativa*. Hence, its genome can be helpful to annotate sequences of *Z*. *mays* and *S*. *bicolor* genomes. Furthermore, the motif analysis discovered the presence of additional conserved motifs outside bZIP, BBR, and BZR domain that may be involved in the proper functioning of proteins. Gene structure gives understanding that the number of exons and introns vary in *T*. *aestivum* genes. The gain or loss of exons/intron may arise during the evolution of these genes. Additionally, prediction of subcellular localization revealed that most of the TFs were localized in the nucleus that is key for efficient functioning of TF genes. Finally, this system biology approach develops a thorough understanding of TabZIP, TaBBR, and TaBZR genes that will contribute for further predicting the function of these genes in *T*. *aestivum*.

The article "Genome-wide analysis of bZIP, BBR, and BZR transcription factors in Triticum aestivum" was retracted in 2022. Reasons: compromised peer review; a conflict of interest; concerns about the authorship.

## Supporting information

S1 Fig Conserved domain analysis of TabZIP proteins. (PPTX)

S2 Fig TabZIP conserved motifs logos using MEME tool. (PPTX)

S3 Fig Conserved motif location of TabZIP proteins using MEME tool. **(A)** Motifs location from TraesCS5A02G440400.1-TraesCS7D02G171300.1. **(B)** Motifs location from TraesCS2A02G245700.2-TraesCS1A02G258100.1. **(C)** Motifs locations from TraesCS1D02G257400.1-TraesCS7D02G268400.1. **(D)** Motifs locations from TraesCS6B02G318700.1-TraesCS5D02G273500.1 **(E)** Motifs Consensus.
(PPTX)

S4 Fig TaBBR/BPC conserved motif logos and location using MEME tool. **(A)** TaBBR/BPC conserved motif logos. **(B)** Conserved motif location of TaBBR/BPC proteins.
(PPTX)

S5 Fig TaBZR conserved motif logos and locations using MEME tool. **(A)** TaBZR conserved motif logos. **(B)** Conserved motif location of TaBZR proteins.
(PPTX)

S6 Fig Subcellular localization of TabZIP Proteins. **(A)** Shows from TaBZIP2-TabZIP30. **(B)** Shows from TaBZIP31-TabZIP45. **(C)** Shows from TaBZIP46-TabZIP84.
(PPTX)

S7 Fig Subcellular localization and gene models of TaBBR Proteins. **(A)** Subcellular localization of TaBBR Proteins. **(B)** Gene model prediction of TaBBR.
(PPTX)

S8 Fig Subcellular localization of TaBZR Proteins. (PPTX)

S9 Fig Gene model prediction of TabZIP. **(A)** Shows from TabZIP2-TabZIP20. **(B)** Shows from TabZIP21-TabZIP40. **(C)** Shows from TabZIP41-TabZIP60. **(D)** Shows from TabZIP61-TabZIP84.
(PPTX)

S1 Table bZIP transcription factor from selected monocots. (XLSX)

S2 Table BBR transcription factor from selected monocots. (XLSX)

S3 Table BZR transcription factor from selected monocots. (XLSX)

S4 Table *Triticum aestivum* bZIP subcellular localization. (XLSX)

S5 Table *Triticum aestivum* BBR subcellular localization. (XLSX)

S6 Table *Triticum aestivum* BZR subcellular localization. (XLSX)

S1 File (DOCX)

S2 File (DOCX)

S3 File (DOCX)
